# Research on the Application Effect of Strengthening Risk Management in Continuous Renal Replacement Therapy Nursing of Critically Ill Patients

**DOI:** 10.1155/2022/2363877

**Published:** 2022-07-08

**Authors:** Huimei Yang, Yan Chen, Mingxia Fu

**Affiliations:** ^1^Department of Emergency, Hubei University of Medicine, Shiyan, China; ^2^Department of Blood Purification, Hubei University of Medicine, Shiyan, China; ^3^Department of Gastroenterology 3 Ward, Renmin Hospital, Hubei University of Medicine, Shiyan, Hubei 442000, China

## Abstract

**Objective:**

To evaluate the efficacy of risk management in the nursing of critically ill patients on continuous renal replacement therapy (CRRT).

**Methods:**

In this retrospective study, 80 critically ill patients on continuous renal replacement therapy in our hospital from February 2020 to February 2021 were recruited. They were randomly assigned to receive either the risk management treatment (risk management group) or the conventional management treatment (conventional management group) via the random number table method. Outcome measurements included the occurrence of adverse events, complications, psychological status, quality of life, treatment compliance, duration of CRRT, and nursing satisfaction.

**Results:**

Risk management treatment was associated with lower incidence of adverse events compared to conventional management treatment (*P* value < 0.05). The risk management group also resulted in a lower incidence of complications compared to the conventional management group (*P* value < 0.05). Patients who received risk management treatments demonstrated a significantly lower anxiety/depression level and a higher World Health Organization Quality of Life Brief Version (WHOQOL-BREF) (*P* value < 0.05). The risk management group resulted in more cases with high compliance and fewer cases with moderate and poor compliance (*P* < 0.05). Risk management was associated with more cases with a CRRT duration less than 36 hours and 36–48 hours and fewer cases with a duration longer than 48 h (*X*^2^ = 2.999, *P* value < 0.05). Patients who were given a risk management treatment had a higher nursing satisfaction compared to conventional management treatment (*X*^2^ = 4.501, *P* value < 0.05).

**Conclusion:**

Risk management treatment in caring of critically ill patients on CRRT shows better efficacy than conventional management treatments.

## 1. Introduction

Continuous renal replacement therapy (CRRT) is more effective than intermittent hemodialysis therapy in treating critically ill patients. It enables the restoring of renal function and the maintenance of stable blood circulation [1]. CRRT is a blood purification treatment method that uses the principle of convection to perform solute exchange and water removal with slow blood flow rate and/or dialysate flow rate. As the clinical application of CRRT becomes more common, it causes more hidden safety hazards that affect the quality of care. Therefore, managing patients undergoing CRRT treatment poses a challenge for clinical nursing. However, the critical condition and the lengthy duration of treatment bring considerable difficulties in patient care [2]. The patients are predisposed to various complications, such as extracorporeal circulation coagulation and catheter-related infections. Such complications not only adversely affect the therapeutic effect of CRRT but also lead to more frequent occurrence of negative emotions in patients [3]. CRRT is an invasive treatment and mainly targets critically ill patients. Also, the treatment requires a long duration. As a result, continuous anticoagulation treatment is required to ensure the smoothness of cardiopulmonary bypass. In clinical treatment, more nursing risks will inevitably occur. The undergraduate nursing staff usually lacks experience and has poor critical thinking skills. This may result in patient's conditional changes not detected in time during the CRRT treatment. By applying various risk assessments, nursing staff can better identify risks. All in all, the treatment of such patients requires active care, effective assessment of risk factors, and preventive interventions to effectively control the complications mentioned above [4]. The present study recruited 80 critically ill patients on continuous renal replacement therapy in our hospital from February 2020 to February 2021 to evaluate the efficacy of risk management in on CRRT.

## 2. Materials and Methods

### 2.1. Baseline Data

In this retrospective study, 80 critically ill patients on continuous renal replacement therapy in our hospital were recruited from February 2020 to February 2021. They were assigned randomly either to a risk management group or conventional management group. The baseline characteristics of the risk management group are as follows: aged between 23 and 87 with a mean of 55.23 and standard deviation of 9.58 years, 19 females and 21 males, 11 cases of multiorgan failure, 8 cases of acid-base imbalance, 5 cases of infectious shock, 4 cases of cardiac insufficiency, 3 cases of chronic renal failure, 3 cases of acute renal injury hyperkalemia, 2 cases of acute severe pancreatitis, 2 cases of crush syndrome, and 2 cases of organophosphorus pesticide poisoning. These baseline characteristics are comparable with the conventional management group, which are aged between 24 and 88 years with a mean of 55.85 and a standard deviation of 9.69 years, 18 females and 22 males, 10 cases of multiorgan failure, 9 cases of acid-base imbalance, 6 cases of infectious shock, 3 cases of cardiac insufficiency, 3 cases of chronic renal failure, 3 cases of acute renal injury hyperkalemia, 3 cases of acute severe pancreatitis, 2 cases of crush syndrome, and 1 case of organophosphorus pesticide poisoning (*P* value > 0.05). This study was approved by the ethics committee of Renmin Hospital, Hubei University of Medicine, Approval No. 7/337917. All patients and their families were onboard with informed consent.

#### 2.1.1. Inclusion Criteria

(1) Symptoms of water overload, oliguria, and increased creatinine; (2) indications for CRRT; (3) acute physiology and chronic health score ≥15 points; (4) normal vascular access function; (5) an imbalance of acid-base metabolism; and (6) combined electrolyte imbalance.

#### 2.1.2. Exclusion Criteria

(1) Intellectual dysfunction; (2) withdrawal of consent halfway; (3) chronic kidney disease in the past; (4) autoimmune diseases such as connective tissue disease, malignant tumor, and systemic lupus erythematosus; and (5) mental disorders.

### 2.2. Treatment Methods

The two groups of patients were also given Chinese enema treatment with the following herbal composition: 30 g each of rhubarb, dandelion, astragalus, salvia, and oyster. The ingredients were soaked in cold water for 30 minutes, then added into 1000 ml of water, and decocted to 200 ml for later use. The elderly took 100 ml of retention enema each time. Those in better conditions took 100 ml of retention enema each time. Before enema, the traditional Chinese medicine was heated to about 40°C. The patients received the herbal treatment one time a day for 7 days.

#### 2.2.1. Conventional Management

The nursing staff assessed patients' acid-base balance, coagulation status, and vascular access before preparing nursing materials and equipment. They prepared relevant nursing items and confirmed patients' conditions and identity. Blood filters and lines were set up for the closed preflush to establish the extracorporeal circulation with prepared vascular access. Later, the central venous indwelling catheter was connected. Then an assessment of blood flow of the central venous indwelling catheter was performed. The patients' conditions were closely monitored during the treatment. They were also actively encouraged to relieve negative feelings. After the treatment, patients were given health education lessons.

#### 2.2.2. Risk Management Group

Nursing risk management protocols were formulated. A nursing risk management team was established, including attending physicians, head nurses and their assistants, and full-time duty nurses. A closed-loop nursing risk management model for CRRT was then developed. First, the nursing risk factors were retrieved from Wanfang and CNKI databases. Then records from previous clinical nursing experience were summarized. The nursing risk management model was formulated followed by intergroup training. The team members screened relevant information to prevent potential nursing risk factors. An early warning mechanism for nursing risk factors, a standardized treatment process, and a contingency plan after exposure to critical complications were established. Risk management was conducted according to the “ADQI Consensus: Patient and Practical Choices in Continuous Renal Replacement Therapy” [5].

(1) Prevention of hypotension: in order to prevent hypotension, strengthen the attention span of the monitoring alarm. Timely intervene on the occurrence of blood pressure changes. Additionally, make reasonable arrangements on the order of fluid input. Accurately record the input time on the record sheet to ensure that the liquid is dripped in a timely and standardized manner. For patients with severe hypoalbuminemia, strengthen dehydration treatment if necessary. Input the albumin shortly after getting on the machine to increase the colloid osmotic pressure. As such, the renal replacement therapy process can be stably ultrafiltrationally dehydrated. This improves the treatment effect and prevents the occurrence of low blood pressure. (2) To prevent hypoglycemia, the bedside blood glucose monitoring sheet was used. According to the guidelines of the American Society of Endocrinology on blood glucose control [6], a standardized template was formulated, a form record sheet was made, and blood glucose was monitored regularly. Timely flush the speed of insulin pump to reduce the occurrence of hypoglycemia. (3) Prevention of coagulation. The whole department conducted training on standardizing the collection method and the collection site of blood samples. They also conducted the homogenization management of blood sample collection to ensure the accuracy of the results. The quantity of anticoagulant drugs was adjusted in time based on the results. (4) Prevention of central venous catheter-related bloodstream infection. A central venous indwelling catheter is a safety hazard for CRRT patients. This is because catheter-related bloodstream infection is the most serious complication of central venous catheterization. Therefore, the skin condition of the puncture point should be observed on a daily basis. If symptoms such as redness, swelling, and exudation of the puncture site are found, report and deal with them immediately. Maintain hand hygiene according to standardized procedures. Nursing staff must strictly implement aseptic operations during the process of dispensing and replacing liquids, and disinfect the interface to prevent the occurrence of iatrogenic infection. When the patient has an unexplained rise in body temperature, blood samples should be collected as soon as possible for culture.

### 2.3. Outcome Measurements

1. The occurrence of risk factors was recorded.
2. The occurrence of complications was recorded.
3. Psychological status and quality of life. Anxiety and depression self-rating scales and the World Health Organization Quality of Life Brief Version (WHOQOL-BREF) were used to evaluate the psychological status and life quality of patients, with a total score of 0 to 100 points. The score of the anxiety and depression scales was proportional to the severity of the anxiety and depression. A higher WHOQOL-BREF score directly results in a better quality of life [7, 8]. WHOQOL-BREF includes physical health, mental state, independent ability, social relations, personal beliefs, and surrounding environment in six areas and 24 aspects. All areas and aspects are quantified in a way that a higher total score indicates a better the quality of life.
4. Treatment compliance. Complete cooperation, occasional cooperation, and uncooperativeness were considered as high, moderate, and poor compliance, respectively.
5. Treatment compliance was judged from four aspects: whether the patient goes to hospital for CRRT on time, whether the patient takes medicine as prescribed, whether the patient comes for follow-up and medical checkup regularly, and whether the patient contacts the doctor in time. According to the patient's treatment record sheet, complete cooperation (high) means that the patient fully complies with the four rules mentioned above. Occasional cooperation (moderate) means the patient fails to comply with any of the four aforementioned rules more than once. Noncooperation (poor) means the patient fails to comply with the any of the four aforementioned rules more than three times.
6. The CRRT duration was recorded.
7. Nursing satisfaction. The patient's degree of satisfaction with nursing was assessed using a self-made nursing satisfaction questionnaire carrying 10 points. The scores of 0–2 points, 3–5 points, 6–8 points, and 9–10 points represent dissatisfied, moderately satisfied, satisfied, and highly satisfied, respectively.

### 2.4. Statistical Analysis

SPSS 20.0 was used for data analysis. The measurements were expressed as ($\bar{x}\pm s$) and processed using the *t*-test. The counts were expressed as the number of cases (rate) and analyzed using the chi-square analysis. The rank-sum test was used to compare scaled value. Differences were considered as statistically significant if *P* value < 0.05.

## 3. Results

### 3.1. Risk Factors

Risk management led to a significantly lower occurrence of risk factors (5.00% [2/40]) versus conventional management (25.00% [10/40]) (*X*^2^ = 6.275, *P*=0.012) (Table 1).

### 3.2. Complications

Risk management resulted in a lower incidence of complications (10.00% [4/40]) versus conventional management (30.00% [12/40]) (*X*^2^ = 5.000, *P*=0.025) (Table 2).

### 3.3. Psychological Status and Quality of Life

Before the intervention, two groups demonstrated similar anxiety scores, depression scores, and World Health Organization Quality of Life Brief Version (WHOQOL-BREF) scores (*P* > 0.05). Patients who received the risk management treatment showed a significantly lower anxiety and depression scores and a higher WHOQOL-BREF score versus patients who received the conventional management treatment (*P* < 0.001) (Table 3).

### 3.4. Treatment Compliance

Before the intervention, the two groups did not differ in terms of treatment compliance (*P* value > 0.05). Risk management resulted in more cases with high compliance and fewer cases with moderate and poor compliance (*P* < 0.05) (Table 4).

### 3.5. CRRT Duration

Risk management resulted in more cases with a CRRT duration shorter than 36 hours and 36–48 hours and fewer cases with a duration longer than 48 hours (*Z* = 2.999, *P*=0.003) (Table 5).

### 3.6. Nursing Satisfaction

Patients receiving risk management had a higher nursing satisfaction (92.50% [37/40]) versus conventional management (75.00, [30/40]) (*X*^2^ = 4.501, *P*=0.034) (Table 6).

## 4. Discussion

Continuous renal replacement therapy is a blood purification technique commonly used in the treatment for critically ill patients. This therapy can remove solutes continuously and support organ function [5, 6]. During the treatment, CRRT removes inflammatory factors tremendously and maintains hemodynamic balance in the kidney. It also reduces the possibility of ischemia to promote the balance of the patient's internal environment and benefits a longer lifespan. However, intermittent hemodialysis, which is also a type of renal replacement therapy, only aims at relieving pain. It has a large deficiency in maintaining the internal environment of body and the overall effect is relatively poor. Currently, CRRT is mostly used for systemic severe diseases, such as systemic inflammatory response syndrome, multiple organ dysfunction syndrome, adult respiratory distress syndrome, and severe acute pancreatitis. Patients in this study have multiple organ failure, acid-base imbalance, infectious shock, cardiac insufficiency, acute severe pancreatitis, and organophosphorus pesticide poisoning. To implement CRRT and provide specialized care to critically ill patients, CRRT-specialized nurses are required to be present throughout [9, 10] the treatment. In recent years, clinical application of CRRT has become increasingly sophisticated. However, with the invasive nature of CRRT, the long duration of the treatment and the need for continuous anticoagulation to ensure the potency of extracorporeal circulation results in a high incidence of nursing risks in its clinical practice [11, 12]. For such patients, nursing risk management provides effective control of various risk factors and considerably reduces the occurrence of complications. It also alleviates negative feelings and improves their quality of life [13, 14]. This study incorporates Chinese medicine enema adjuvant therapy that can improve the efficacy of patients with acute kidney injury. Chinese medicine enema is easy to operate and is absorbed quickly. Thus, it can effectively reduce the stimulation of the gastrointestinal tract caused the bitterness and coldness of the drug. According to the Chinese history of medicine, renal injury is in the category of “kidney wind, stagnation.” Toxic and blood stasis syndrome should be treated by detoxification to remove blood stasis and invigorate the organ [10]. The herbs used in traditional Chinese medicine enema are mainly rhubarb, dandelion, astragalus salvia, and oyster. Among them, rhubarb is mainly used as a laxative. It cools and detoxifies the blood. It removes the stasis and then activates the blood. Salvia can activate blood and remove blood stasis. Oysters are astringent. It relieves rhubarb's effect on diarrhea. Combination of various herbs achieves detoxification and removal of blood stasis. Such combination also invigorates the organ and leads to diuresis. Pharmacological research shows that [11] rhubarb has a significant diuretic effect. It also improves renal function and inhibits a variety of Gram-negative and Gram-positive bacteria, thus improving blood rheology. The present study shows that risk management leads to a significantly lower occurrence of risk factors and complications versus conventional management. Moreover, it helps patients to achieve significantly lower anxiety and depression scores and higher WHOQOL-BREF scores versus conventional management. Perhaps the assessment and individualized control of risk factors in nursing risk management can effectively eliminate patients' negative feeling and thus improve their quality of life [15–17]. Furthermore, risk management results in more cases with high compliance with a CRRT duration shorter than 36 hours and 36–48 hours versus conventional management. This may be attributed to the fact that nursing risk management effectively prevents treatment-related risk factors and enhances the safety of treatment. Thus, it can effectively improve the outcomes and patients' satisfaction [18, 19].

Professional nursing aims to provide continuous, holistic, and personalized care to achieve desired nursing outcomes. Therefore, a detailed care plan covering the whole process is necessary to control and quantitatively assess CRRT. It addresses malfunctions in extracorporeal circulation and thus minimizes the risk of care to ensure its safety and continuity. To sum up, risk management treatments in the care of critically ill patients on CRRT show better efficacy than conventional management treatment.

## Figures and Tables

**Table 1:** Comparison of adverse risk events (*n* (%)).

Groups	*n*	Tube dislodgement	Catheter-associated infection	Extracorporeal circulation coagulation	Others	Incidence
Risk management group	40	0 (0)	1 (2.50)	1 (2.50)	0 (0)	2 (5.00)
Conventional management group	40	2 (5.00)	2 (5.00)	4 (10.00)	2 (5.00)	10 (25.00)
*χ* ^2^						6.275
*P* value						0.012

**Table 2:** Comparison of complications (*n* (%)).

Groups	*n*	Hemorrhage	Coagulation	Hypoglycemia	Hypotension	Incidence
Risk management group	40	1 (2.50)	1 (2.50)	1 (2.50)	1 (2.50)	4 (10.00)
Conventional management group	40	5 (12.50)	4 (10.00)	2 (5.00)	1 (2.50)	12 (30.00)
*χ* ^2^						5.000
*P* value						0.025

**Table 3:** Comparison of psychological status and quality of life (points, $\bar{x}\pm s$).

Time points	Groups	*n*	Anxiety scores	Depression scores	WHOQOL-BREF scores
Before intervention	Risk management group	40	52.70 ± 5.80	53.31 ± 5.80	58.62 ± 9.23
	Conventional group	40	52.51 ± 5.67	53.22 ± 5.70	59.02 ± 9.13
*t*-value			0.148	0.070	0.195
*P* value			0.883	0.944	0.846

After intervention	Risk management group	40	45.20 ± 4.50	43.22 ± 3.97	77.25 ± 9.32
	Conventional group	40	49.81 ± 4.68	46.96 ± 4.68	68.12 ± 9.14
*t*-value			4.491	3.854	4.424
*P* value			<0.001	<0.001	<0.001

**Table 4:** Comparison of treatment compliance ($\bar{x}\pm s$).

Time points	Groups	*n*	High	Moderate	Poor
Before intervention	Risk management group	40	28 (70.00)	6 (15.00)	6 (15.00)
	Conventional management group	40	29 (72.50)	6 (15.00)	5 (12.50)
*Z*-value				0.278	
*P* value				0.781	

After intervention	Risk management group	40	37 (92.50)	2 (5.00)	1 (2.50)
	Conventional management group	40	30 (75.00)	5 (12.50)	5 (12.50)
*Z*-value				2.115	
*P* value				0.035	

**Table 5:** Comparison of CRRT duration (*n* (%)).

Groups	*n*	<36 h	36 ∼ 48 h	>48 h
Risk management group	40	7 (17.50)	27 (67.50)	6 (15.00)
Conventional management group	40	1 (2.50)	23 (57.50)	16 (40.00)
*Z*			2.999	
*P* value			0.003	

**Table 6:** Comparison of nursing satisfaction (*n* (%)).

Groups	*n*	Highly satisfied	Satisfied	Moderately satisfied	Dissatisfied	Satisfaction
Risk management group	40	32 (80.00)	5 (12.50)	2 (5.00)	1 (2.50)	37 (92.50)
Conventional management group	40	27 (67.50)	3 (7.50)	7 (17.50)	3 (7.50)	30 (75.00)
*χ* ^2^						4.501
*P* value						0.034

## Data Availability

All data generated or analyzed during this study are included in this published article.
